The article "Xingnao Kaiqiao Acupuncture Combined with Butylphthalide Sodium Chloride Injection in the Treatment of Acute Cerebral Infarction and Its Effect on the Levels of Serum Malondialdehyde, Superoxide Dismutase, and Glutathione Peroxidase" was published in 2022. Journal: Evid Based Complement Alternat Med.

# Xingnao Kaiqiao Acupuncture Combined with Butylphthalide Sodium Chloride Injection in the Treatment of Acute Cerebral Infarction and Its Effect on the Levels of Serum Malondialdehyde, Superoxide Dismutase, and Glutathione Peroxidase

**DOI:** 10.1155/2022/5990203

**Published:** 2022-08-26

**Authors:** Junyi Cui, Handi Jia

**Affiliations:** ^1^Department of Neurology, The People's Hospital of Suzhou New District, Suzhou, China; ^2^Department of Chinese Medicine, The People's Hospital of Suzhou New District, Suzhou, China

## Abstract

**Objective:**

The aim of this study is to explore the therapeutic effect of Xingnao kaiqiao acupuncture combined with butylphthalide sodium chloride injection on acute cerebral infarction and its effect on the levels of serum malondialdehyde (MDA), superoxide dismutase (SOD), and glutathione peroxidase (GSH).

**Methods:**

120 patients with acute cerebral infarction who were treated in our hospital from March 2020 to March 2022 and met the inclusion and exclusion criteria were divided into two groups. The control group was treated with sodium butylphthalide chloride injection, and the study group was treated with Xingnao kaiqiao acupuncture combined with sodium butylphthalide chloride injection.

**Results:**

After treatment, the levels of neurotransmitters, the TTP and RI and MDA in both groups decreased, and the Qmean, CBV values, and the levels of SOD and GSH increased, and the changes of index in the study group were more significant than those in the control group (*P* < 0.05). After treatment, the NIHSS score and syndrome score of the two groups decreased, the MMSE score increased, the NIHSS score and syndrome score of the study group decreased more significantly than that of the control group, and MMSE score increased more significantly than that of the control group (*P* < 0.05). In terms of clinical efficacy, the total effective rate of the study group was higher than that of the control group (*P* < 0.05).

**Conclusion:**

Xingnao kaiqiao acupuncture combined with butylphthalide sodium chloride injection is effective in patients with acute cerebral infarction. It can improve the level of neurotransmitters and cerebral blood flow perfusion and inhibit the abnormal expression of MDA, SOD, and GSH.

## 1. Introduction

Acute cerebral infarction, also known as ischemic stroke, refers to cerebral ischemia and hypoxia caused by insufficient blood supply of internal carotid artery or vertebrobasilar artery, resulting in focal brain tissue necrosis and softening, and then corresponding neurological symptoms, including cerebral thrombosis, lacunar infarction, cerebral embolism, etc., which is the most common cerebrovascular disease. After the occurrence of the disease, patients are mostly accompanied by symptoms of varying degrees of neurological loss; it seriously threatens the life and safety of patients [1]. The incidence of cerebral infarction is high, the disability rate is high, about 70% of patients will leave sequelae; in clinical, the abnormal autonomic nerve function caused by cerebral infarction is gradually being paid attention to and studied.

The pathogenesis of acute cerebral infarction is more complex, blood viscosity and platelet aggregation rate increase, cerebral arteriosclerosis makes blood vessels narrower or blocked, and is prone to acute cerebral ischemia and hypoxia necrosis. The risk factors of acute cerebral infarction include age, diabetes, hyperlipidemia, hypertension, obesity, and so on. Timely and effective treatment for patients with acute cerebral infarction is particularly important to improve the clinical efficacy and quality of life of patients and reduce the recurrence rate. In the clinical treatment of acute progressive cerebral infarction, time window and ultraearly thrombolysis are very important. At the same time, anticoagulation, defibrillation, antiplatelet, brain protection, and traditional Chinese and Western medicine are provided according to the condition. The etiology of acute cerebral infarction is complex, which is the result of multifactors and multisystem participation. Therefore, it is necessary to comprehensively use appropriate treatment methods to improve the prognosis of patients, improve clinical efficacy, and reduce the recurrence rate. The key to the treatment of acute cerebral infarction is to recanalize or improve the blood supply of ischemic brain tissue as soon as possible, save the brain cells in the ischemic penumbra, and alleviate the secondary tissue damage caused by ischemia and hypoxia. At present, the traditional treatment for acute cerebral infarction is mainly through the influence of hemodynamics, such as thrombolysis and thrombectomy. However, due to the limitation of “time window” and bleeding risk, many patients have poor efficacy and prognosis.

Butylphthalide is a new chemical drug independently developed in the cerebrovascular field in China. It is a drug extracted from celery seeds. Its main drug active component is the synthetic racemic dl-3-n-butylphthalide. It is a fat soluble drug that can directly exert its efficacy through the human blood-brain barrier. Since 2004, butylphthalide has been widely used in the treatment of acute cerebral infarction and its sequelae [2].

Acute cerebral infarction belongs to the category of “stroke” in traditional Chinese medicine. Traditional Chinese medicine has an ideal effect in the treatment of “stroke” diseases and has a long history [3, 4]. In view of this, this paper analyzes the therapeutic effect of Xingnao kaiqiao acupuncture combined with butylphthalide sodium chloride injection on acute cerebral infarction and analyzes the effect on the level of serum malondialdehyde (MDA), superoxide dismutase (SOD), and glutathione peroxidase (GSH), which are related to oxidative stress.

## 2. Materials and Methods

### 2.1. Research Subjects

120 patients with acute cerebral infarction treated in our hospital from March 2020 to March 2022 were randomly divided into a control group (*n* = 60) and a study group (*n* = 60). Moreover, the informed consent of patients has been obtained. The details of the two groups are shown in Table 1, and the two groups are comparable (*P* > 0.05).

The inclusion criteria were as follows: all patients met the diagnostic criteria of traditional Chinese and Western medicine for acute cerebral infarction in the Chinese guidelines for the diagnosis and treatment of acute ischemic stroke 2018 [5] and the criteria for the diagnosis and efficacy evaluation of stroke [6] and were diagnosed by magnetic resonance imaging. They were hospitalized within 24 hours of onset and first onset within 1 year. They voluntarily participated in this study.

The exclusion criteria were as follows: deceased with previous myocardial infarction; unclear consciousness; persons with mental illness; drug allergy; unable to communicate; and acute and chronic infection.

### 2.2. Treatment

Both groups received routine treatment such as oxygen inhalation after admission. The control group was treated with butylphthalide sodium chloride injection (stone Pharmaceutical Group Enbipu Pharmaceutical Co., Ltd., national drug approval word: h20100041), intravenous drip, 100 ml/time, twice a day, for 2 weeks. On the basis of the control group, the study group was treated with Xingnao kaiqiao acupuncture, with the bilateral Neiguan point, Sanyinjiao point, and Shuigou point on the affected side as the main points, Chize point, Weizhong point, and Jiquan point on the affected side as the matching points, and the Neiguan point was treated with twisting, lifting, and inserting catharsis combined with direct acupuncture for 0.5 inch for 1 minute; the Shuigou point uses the heavy bird pecking technique to obliquely stab 0.5 inch, with tears or wet eyes as the degree; the Sanyinjiao point on the affected side was obliquely stabbed for 1 inch with the upper limb twitch on the affected side as the degree. The method of lifting, inserting, and purging is used to directly stab the Jiquan point for 1 inch, with the degree of upper limb twitch on the affected side. The Chize point is directly stabbed with lifting, inserting, and purging method for 1 inch, and the finger twitch is the degree. The Weizhong point is directly punctured by the lifting, inserting, and purging method for 1 inch, with the degree of twitch of the lower limbs on the affected side. These were done once a day, 6 times a week, continuous treatment for 2 weeks.

### 2.3. Index Observation

#### 2.3.1. Determination of Serum Indexes

3 ml of fasting venous blood was taken before and after treatment, and the neurotransmitter indexes (norepinephrine (NE), dopamine (DA), serotonin (5-HT), epinephrine (E)) and glutathione peroxidase (GSH) were measured by a reeders automatic multifunctional microplate reader. The levels of malondialdehyde (MDA) and superoxide dismutase (SOD) were measured by colorimetry.

#### 2.3.2. Evaluation of Cerebral Blood Flow Perfusion

Before and after treatment, the patients' cerebral blood flow perfusion was evaluated according to the ultrasonic parameters blood flow peak time (TTP), resistance index (RI), average blood flow (Qmean), and cerebral blood volume (CBV).

#### 2.3.3. Neurological, Cognitive, and Syndrome Score Evaluation

The neurological and cognitive functions were evaluated by NIHSS and MMSE before and after treatment. The lowest score of NIHSS was 0 and the highest score was 45. The lower the score, the lighter the neurological deficit. The lowest score of MMSE is 0 and the highest score is 30. The higher the score, the better the cognition. TCM syndromes are evaluated according to the standard for diagnosis and efficacy evaluation of stroke [6]. The higher the score, the more serious the symptoms are.

#### 2.3.4. Clinical Efficacy Evaluation

The clinical efficacy of patients is evaluated according to the NIHSS score value, in which the decrease of NIHSS score value ≥ 45% is significant, 18% ≤ NIHSS score value < 45% is improvement, and it is invalid if it fails to meet the above standards.

#### 2.3.5. Adverse Reaction Evaluation

The adverse reactions of the two groups were evaluated, including retching, nausea, dry mouth, abdominal distension, headache, and so on.

### 2.4. Statistical Analysis

SPSS 22.0 software was used for data analysis. The measurement data conforming to the normal distribution were described by$\left(\bar{x}\pm s\right)$, independent sample *t* test was performed between the two groups, and paired *t* test was performed within the group. The counting data were expressed by frequency and percentage, and the comparison between groups was expressed by frequency *χ*^2^. In the test, *P* < 0.05 indicates that the difference is statistically significant and *P* < 0.001 indicates that the difference is statistically significant.

## 3. Results

### 3.1. Comparison of Neurotransmitter Levels between the Two Groups before and after Treatment

The comparison of NE, DA, 5-HT, and *E* indexes between the two groups before and after treatment showed that the comparison of various indexes between the two groups before treatment was meaningless (*P* > 0.05). After treatment, the levels of various indexes in the two groups decreased and the levels of various indexes in the study group decreased more significantly than those in the control group (*P* < 0.05). See Table 2.

### 3.2. Comparison of Cerebral Blood Flow Perfusion Indexes between the Two Groups before and after Treatment

The comparison of cerebral blood flow perfusion indexes between the two groups before and after treatment showed that the comparison of cerebral blood flow perfusion indexes between the two groups before treatment was meaningless (*P* > 0.05). After treatment, the TTP and RI values of the two groups decreased, and the Qmean and CBV values increased. The TTP and RI values of the study group decreased more significantly than those of the control group, and the Qmean and CBV values increased more significantly than those of the control group (*P* < 0.05). See Table 3.

### 3.3. Comparison of MDA, SOD, and GSH Index Levels between the Two Groups before and after Treatment

The comparison of MDA, SOD, and GSH index levels between the two groups before and after treatment showed that the comparison of various index levels between the two groups before treatment was meaningless (*P* > 0.05). After treatment, the levels of SOD and GSH increased and the level of MDA decreased in the two groups, and the levels of SOD and GSH in the study group increased more significantly than those in the control group and the level of MDA decreased more significantly than those in the control group (*P* < 0.05). See Table 4.

### 3.4. Comparison of the NIHSS, MMSE Score, and Syndrome Score between the Two Groups before and after Treatment

The comparison of the NIHSS, MMSE score and syndrome score between the two groups before and after treatment showed that the comparison of various scores between the two groups before treatment was meaningless (*P* > 0.05). After treatment, NIHSS score and syndrome score of the two groups decreased, MMSE score increased, NIHSS score and syndrome score of the study group decreased more significantly than that of the control group and the MMSE score increased more significantly than that of the control group (*P* < 0.05). See Table 5.

### 3.5. Comparison of Clinical Efficacy between the Two Groups

In terms of clinical efficacy, the total effective rate of the study group was higher than that of the control group (*P* < 0.05). See Table 6.

### 3.6. Occurrence of Adverse Events during  Treatment in the Two Groups

There was no significant difference in the incidence of adverse events between the two groups (*P* > 0.05). See Table 7.

## 4. Discussion

Acute cerebral infarction has a high risk of morbidity, and its disability rate and mortality are higher than other brain diseases, which seriously affects the quality of life of patients. At present, the pathogenesis of the disease is not clear and there is no specific scheme to treat the disease [7]. At present, butylphthalide has been widely used in the treatment of patients with acute cerebral infarction. According to research [8, 9], it can promote the expression of prostaglandins by inhibiting the activity of arachidonic acid, inhibit the decrease of intracellular Ca^2+^ content, restore cerebral blood supply, improve local microcirculation, and play a role in the treatment of diseases by inhibiting excessive free radicals. From the study, we found that single drug butylphthalide sodium chloride injection cannot achieve the expected effect.

Butylphthalide has multiple pharmacological effects. It can improve the neurological deficit and prognosis of acute cerebral infarction by reconstructing cerebral ischemia microcirculation, inhibiting neuronal apoptosis, protecting mitochondria, scavenging free radicals, antiplatelet aggregation, inhibiting thrombosis, reducing inflammatory reaction, and protecting vascular endothelial cells. The results showed that butylphthalide could reduce the levels of IL-6, IL-8, CRP, and TNF in serum of patients with acute cerebral infarction-*α*-expression of inflammatory factors such as Lp-PLA2 and hs-CRP, decrease serum endothelin, TXA2FIB, DDI, TXB2, Pai-1 level, antiplatelet aggregation, inhibit thrombosis, improve hypercoagulable state, reduce the size and thickness of carotid plaque, increase the number of circulating endothelial progenitor cells in serum, and enhance their migration ability to the injured area.

Due to the advantages of high safety and excellent effect of traditional Chinese medicine, it has become the focus of clinical attention. Traditional Chinese medicine believes that deficiency of qi and blood is the disease pathogenesis of acute cerebral infarction. In the process of onset, combined with the influence of wind, fire, phlegm, and blood stasis, it eventually leads to the disorder of qi and blood and the imbalance of yin and yang [10]. At present, the means of TCM in treating acute cerebral infarction include decoction and acupuncture. Xingnao kaiqiao acupuncture can play a role in the symptoms of stroke. It can promote coma recovery and dredge the meridians. The acupoints are selected according to the pathogenesis of acute cerebral infarction, with the bilateral Neiguan point, affected Sanyinjiao point, and Shuigou point as the main acupoints, and the Chize point, Weizhong point, and Jiquan point on the affected side as the matching points. Among them, acupuncture at the Neiguan point can play the role of xinnao kaiqiao. Acupuncture at the Sanyinjiao point can play the role of dredging collaterals and regulating qi and blood. Acupuncture at the Shuigou point can play the role of kuanxiong liqi. In addition, manipulation and needle feeding control are applied in the process of acupuncture, so as to play a role in the treatment of diseases [11–13]. The results of this study show that on the basis of the treatment of patients with sodium butylphthalide chloride injection, Xingnao kaiqiao acupuncture is added. The results show that the symptoms of such patients are improved most significantly, which can significantly improve the neurological deficit and cognitive impairment and improve the abnormal cerebral blood flow perfusion. The effect is ideal.

The main symptom of acute cerebral infarction is the abnormal expression of neurotransmitter related indicators. The brain injury of patients gradually aggravates during the occurrence of the disease [14, 15]. The results showed that the levels of neurotransmitters such as NE, DA, 5-HT, and *E* in the study group decreased more than those in the control group after treatment. The results suggested that Xingnao kaiqiao acupuncture combined with butylphthalide sodium chloride injection could repair brain injury and inhibit brain injury in patients with acute cerebral infarction, which showed that the levels of neurotransmitters such as NE, DA, 5-HT, and *E* decreased.

Research shows that [16, 17], oxidative stress runs through the whole pathogenesis of acute cerebral infarction. After brain injury and ischemia, a large number of free radicals are accumulated in cells. With the progress of the disease, the number of free radicals increases sharply, and the related enzymes required to remove free radicals cannot be supplemented in time, resulting in the decline of their activity, the disorder of oxidation/antioxidant dynamic balance, resulting in the aggravation of brain injury. At present, it is clinically believed that indicators related to oxidative stress such as MDA, SOD, and GSH are involved in the occurrence of acute cerebral infarction. MDA with increased content in acute cerebral infarction is the degradation product of lipid peroxidation. Its content increases in acute cerebral infarction and the content of SOD and GSH decreases. Therefore, monitoring the level of appeal indicators can evaluate the degree of oxidative stress and reflect the disease status of patients [18–20]. Therefore, in this study, the changes of the abovementioned indexes of the two groups were compared and analyzed. The results showed that the indexes of patients treated with Xingnao kaiqiao acupuncture combined with butylphthalide sodium chloride injection were significantly improved. This result shows that the combination of the two can treat both symptoms and symptoms and repair brain injury by inhibiting oxidative stress.

## 5. Conclusion

The expected effect of Xingnao kaiqiao acupuncture combined with butylphthalide sodium chloride injection in patients with acute cerebral infarction is ideal. It can improve the level of neurotransmitters and inhibit the abnormal expression of MDA, SOD, and GSH.

## Figures and Tables

**Table 1:** General information.

Constituencies	Male/female (example)	Average age (years)	Average time from onset of illness to hospitalization (h)	Lesion site (lobe/basal ganglia/brainstem)	Hyperlipidemia	Hypertension	Diabetes
Control group (*n* = 60)	25/35	52.46 ± 3.75	10.15 ± 1.53	15/30/15	10	9	13
Study group (*n* = 60)	29/31	53.12 ± 3.48	10.18 ± 1.46	16/28/16	12	8	11
*χ * ^2^/*t*	0.539	0.999	0.110	0.134	0.223	0.069	0.208
*P*	0.463	0.320	0.913	0.935	0.637	0.793	0.648

**Table 2:** Comparison of neurotransmitter levels before and after treatment between the two groups (($\bar{x}\pm s$), ng/mL).

Constituencies	*NOT*		*OF*		*5-HT*		*AND*	
	Before treatment	After treatment	Before treatment	After treatment	Before treatment	After treatment	Before treatment	After treatment
Control group (*n* = 60)	109.15 ± 15.03	89.37 ± 12.65	337.15 ± 33.15	279.15 ± 27.62	386.55 ± 37.85	296.17 ± 28.51	33.42 ± 5.96	28.27 ± 4.05
Study group (*n* = 60)	109.47 ± 15.11	59.15 ± 9.62^*∗∗*^	336.89 ± 33.58	203.07 ± 19.26^*∗∗*^	385.63 ± 36.75	229.26 ± 21.37^*∗∗*^	33.60 ± 5.68	20.65 ± 3.11^*∗∗*^
*t*	0.116	14.730	0.043	17.500	0.135	14.550	0.169	11.560
*P*	0.908	0.001	0.966	0.001	0.892	0.001	0.866	0.001

**Table 3:** Comparison of cerebral blood flow perfusion indices before and after treatment between the two groups ($\bar{x}\pm s$).

Constituencies	*TTP (s)*		*Qmean (cm/s)*		*CBV (mL/100 mg)*		*Re*	
	Before treatment	After treatment	Before treatment	After treatment	Before treatment	After treatment	Before treatment	After treatment
Control group (*n* = 60)	128.52 ± 11.26	98.34 ± 10.93	8.12 ± 0.43	9.47 ± 0.42	75.85 ± 6.95	83.05 ± 7.78	0.56 ± 0.14	0.50 ± 0.05
Study group (*n* = 60)	128.68 ± 11.29	74.45 ± 8.65^*∗∗*^	8.15 ± 0.51	10.35 ± 0.26^*∗∗*^	76.10 ± 6.98	92.70 ± 8.31^*∗∗*^	0.59 ± 0.18	0.45 ± 0.03^*∗∗*^
*t*	0.078	13.280	0.348	13.800	0.197	6.566	1.019	6.642
*P*	0.938	0.001	0.728	0.001	0.844	0.001	0.310	0.001

**Table 4:** Comparison of MDA, SOD, and GSH levels before and after treatment ($\bar{x}\pm s$).

Constituencies	*MDA (nmoI/ml)*		*SOD (U/mL)*		*GSH (μmol/L)*	
	Before treatment	After treatment	Before treatment	After treatment	Before treatment	After treatment
Control group (*n* = 60)	7.72 ± 1.81	5.66 ± 0.43	85.16 ± 9.83	97.69 ± 8.79	28.48 ± 5.75	63.75 ± 6.03
Study group (*n* = 60)	7.63 ± 1.12	4.56 ± 0.27^*∗∗*^	85.27 ± 9.14	105.53 ± 10.18^*∗∗*^	29.05 ± 5.43	73.69 ± 7.14^*∗∗*^
*t*	0.078	16.780	0.063	4.515	0.558	8.239
*P*	0.912	0.001	0.949	0.001	0.578	0.001

**Table 5:** Comparison of NIHSS and MMSE scores before and after treatment between the two groups (($\bar{x}\pm s$), score).

Constituencies	*NIHSS*		*MMSE*		*Waiting points*	
	Before treatment	After treatment	Before treatment	After treatment	Before treatment	After treatment
Control group (*n* = 60)	5.62 ± 1.22	3.65 ± 0.78	21.99 ± 5.31	23.54 ± 5.71	15.66 ± 2.15	11.87 ± 1.33
Study group (*n* = 60)	5.64 ± 1.25	2.06 ± 0.45^*∗∗*^	22.04 ± 5.42	25.67 ± 5.91^*∗∗*^	15.76 ± 2.31	9.07 ± 1.12^*∗∗*^
*t*	0.088	13.680	0.051	2.008	0.246	12.470
*P*	0.929	0.001	0.959	0.047	0.807	0.001

**Table 6:** Comparison of clinical efficacy between the two groups (case (%)).

Constituencies	Effective	Improved	Void	Total effectiveness (%)
Control group (*n* = 60)	19	31	10	50 (83.33)
Study group (*n* = 60)	35	22	3	57 (95.00)^*∗∗*^
*χ* ^2^				4.227
*P*				0.040

**Table 7:** Occurrence of adverse events during treatment in two groups (case (%)).

Constituencies	Dry mouth	Abdominal distension	Headache	Dry vomiting, nausea	Total incidence (%)
Control group (*n* = 60)	0	1	1	1	3 (5.00)
Study group (*n* = 60)	2	2	1	2	7 (11.66)
*χ* ^2^					1.745
*P*					0.186

## Data Availability

The data used to support this study are available from the corresponding author upon request.

## References

[1] Edwards M. D., Hughes T. A. T. (2021). Managing blood pressure in acute cerebral infarction. *Journal of Neurology*.

[2] Niu H., Zhang Z., Wang H. (2016). The impact of butylphthalide on the hypothalamus-pituitary-adrenal axis of patients suffering from cerebral infarction in the basal ganglia[J]. *Electronic Physician*.

[3] Ding Y., Xing F. (2021). Research progress in the treatment of acute cerebral infarction by traditional Chinese medicine[J]. *Chinese Journal of Traditional Chinese Medicine Emergency*.

[4] Li Y. (2016). Zhang Lunzhong Research progress in the treatment of acute cerebral infarction by open-end method. *Journal of Cardiovascular and Cerebrovascular Diseases in Integrative Traditional and Western Medicine*.

[5] Branch of Chinese Medical Association N. (2018). Cerebrovascular disease group of neurology branch of Chinese medical association guidelines for the diagnosis and treatment of acute ischemic stroke in China 2018. *Chinese Journal of Neurology*.

[6] (1996). Criteria for diagnosis and efficacy evaluation of stroke disease (trial implementation). *Journal of Beijing University of Traditional Chinese Medicine*.

[7] Yuan T., Wang J. (2021). Clinical and imaging features of acute cerebral infarction in non-small cell lung cancer patients with trousseau syndrome. *Zhongguo Fei Ai Za Zhi*.

[8] Wo X., Han J., Wang J., Wang X., Liu X., Wang Z. (2020). Sequential butylphthalide therapy combined with dual antiplatelet therapy in the treatment of acute cerebral infarction. *Pakistan Journal of Medical Sciences*.

[9] Qian J., Pei Q., Jing R. (2022). Effects of butylphthalide on the levels of serum C-reactive protein, Parkinson disease protein 7 and neurotrophin-3 and neurological function in patients with acute cerebral infarction. *Pakistan Journal of Pharmaceutical Sciences*.

[10] Jia C., Zhang Q., Tao H. (2020). Efficacy of brain-opening acupuncture combined with alteplase in the treatment of acute cerebral infarction and its effect on thromboelastogram index and neurotransmitters. *Shanghai Journal of Acupuncture*.

[11] Wen K., Zhu H., Yuan H. (2016). Effects of different application timings of the brain-opening acupuncture method on cognitive dysfunction in patients with acute cerebral infarction. *Modern Journal of Integrative Medicine*.

[12] Sheng F. (2019). Clinical efficacy of salvia miltiorrhiza polyphenolic acid combined with cerebral glycoside carnosine in the treatment of acute cerebral infarction and its effect on serum GFAP, PAF and MCP-1. *Chinese and Foreign Medical Research*.

[13] Wang H., Fang L., Tan Z. (2017). Effects of brain-opening acupuncture on cognitive function, motor function and nerve function in patients with acute cerebral infarction. *Shanghai Journal of Acupuncture*.

[14] Chang H., Chen Y., Xing H. (2021). Effect of active blood stasis soup on intracranial hemodynamics and serum neurotransmitters in patients with acute cerebral infarction. *Shaanxi Journal of Traditional Chinese Medicine*.

[15] Wang Y., Feng S., Jin H. (2021). Effect of butophthalein combined with atorvastatin calcium on serum inflammatory factors and brain neurotransmitters in patients with acute cerebral infarction. *Clinical Journal of Practical Hospitals*.

[16] Zheng M., Wang X., Yang J., Ma S., Wei Y., Liu S. (2020). Changes of complement and oxidative stress parameters in patients with acute cerebral infarction or cerebral hemorrhage and the clinical significance. *Experimental and Therapeutic Medicine*.

[17] Liu H., Wu X., Luo J. (2020). Adiponectin peptide alleviates oxidative stress and NLRP3 inflammasome activation after cerebral ischemia-reperfusion injury by regulating AMPK/GSK-3*β*. *Experimental Neurology*.

[18] Chun Y., Xu L. (2022). Wan Chunxiao Correlation between expression of oxygenated stress before and after intravenous thrombolysis and functional outcomes in patients with acute cerebral infarction. *Chongqing Medical Journal*.

[19] Zhang H., Zhong C., Wen Z. (2021). Relationship between peripheral blood miR-497 expression and inflammatory oxidative stress in patients with acute cerebral infarction and its predictive value for prognosis. *Journal of Molecular Diagnostics and Treatment*.

[20] Guo Z., Yue Y., Zou Z. (2020). Correlation between serum osteopontin and oxidative stress index levels in the acute stage of acute cerebral infarction and patients with nerve injury and prognosis. *Journal of Clinical and Experimental Medicine*.

